The article "Monitoring and Path Selection of Rural Public Service Environment Based on Data Mining Technology in the New Era" was retracted in 2023. Reasons: signs of a paper mill; suspected computer-generated content; unreliable results or conclusions; concerns about the data.

# Monitoring and Path Selection of Rural Public Service Environment Based on Data Mining Technology in the New Era

**DOI:** 10.1155/2022/1164807

**Published:** 2022-10-06

**Authors:** Shumin Meng

**Affiliations:** Xi'an Jiaotong University, Xi'an 710049, China

## Abstract

The basic public service infrastructure in rural regions now has a lot of issues and flaws, which results in a low efficiency of basic public service delivery and substantially impedes the growth of the rural social economy and the enhancement of farmers' quality of life. Building a smart platform for monitoring the rural public service environment, realising the growth of rural areas, creating a new socialist countryside holistically, and ensuring the sustainable, stable, and healthy development of rural society are all of great strategic importance under the new circumstances. This essay explores ways to further encourage the development of rural public service platforms. In order to choose the best course of action for rural public services in the new era, this study studies the practical problem of rural public services and, using DM (Data Mining) technology, mines the user characteristics of public service platforms. The experimental findings demonstrate that the algorithm's accuracy is 94.38%. With the use of this technique, rural public services may efficiently mine user characteristics and offer specific technical support in the modern day. Decision-makers from all walks of life have an extraordinary desire for information concealed in huge amounts of data in the information age. The advantages of combining the two are becoming more widely recognised.

## 1. Introduction

Rural public service is a very new and important subject. For a long time, China's rural public management and public services are mainly realized by township government organizations and township institutions [1]. From the rural situation, the serious imbalance in the supply of public services between urban and rural areas makes it difficult for rural residents, especially rural poor groups, to obtain basic public services, which leads to their basic right to subsistence and development not being guaranteed, which directly limits the overall improvement of rural population quality [2]. Rural public service, which is a crucial component of government work, is a specific nonexclusive and noncompetitive social service to meet the needs of farming, rural development, or farmers' production and daily lives. It is a form of rural public product that takes the form of labour services, agricultural information, or agricultural technology [3]. The growth of the rural economy, the sustainability of agriculture, and the raising of farmers' living conditions are all directly tied to accelerating the construction of the rural public service platform [4]. The rapid advancement of computer technology and networks has made it possible for an increasing number of people to learn about their social interactions and behaviours with others from the data and from the information sharing and exchange in the traditional information era to the brand-new big data era. To comprehend public opinion and social dynamics, government public departments can also employ the big data analysis of mobile Internet.

The article "Monitoring and Path Selection of Rural Public Service Environment Based on Data Mining Technology in the New Era" was retracted in 2023. Reasons: signs of a paper mill; suspected computer-generated content; unreliable results or conclusions; concerns about the data.

Public service can boost economic growth, increase production efficiency, and provide a strong framework for the complete and coordinated development of rural economies and cultural endeavours [5]. Besides, the rural public services driving the improvement of production efficiency can directly increase farmers' income, the effective supply of convenient transportation, cheap and convenient medical care, education, and other public services can also reduce farmers' living costs and increase farmers' income in disguise. One of the objectives of creating a harmonious socialist society is the reconstruction of rural basic public service platforms, which may foster social fairness and justice, uphold social harmony and stability, and guarantee that everyone shares in the benefits of development [6]. Between the supply of public goods or services in urban and rural areas, there is a significant mismatch. With the Internet's quick development, network resources are multiplying and the volume of network data is growing to the point where every user is faced with an ocean of data. The term “data mining” (DM) [7] refers to the analysis of the microscopic features of the database's data, from which we can derive some macroscopic and macroscopic information that can reflect its features. In order to condense a big amount of data, it is used in the discovery of items' commonality. The public service platform's operation will produce a lot of user-related data, which can be utilised to identify users' access habits using DM or WebDM technology and shorten the time it takes to find resources and services. This article examines the user characteristics of the public service platform, evaluates the situation that rural public service is actually in according to DM technology, and then proposes a course for rural public service in the new era.

It is nevertheless undeniable that the government's provision of rural public amenities in China is insufficient as of the current stage of economic development [8]. The path of rural public service platform building must be improved because it will have a significant impact on the growth of China's rural economy and society as well as the creation of new rural areas [9]. Rebuilding the fundamental public service infrastructure in rural regions has emerged as the institutional safeguard for enacting the urgently needed yet deeply ingrained concept of scientific progress.

The article "Monitoring and Path Selection of Rural Public Service Environment Based on Data Mining Technology in the New Era" was retracted in 2023. Reasons: signs of a paper mill; suspected computer-generated content; unreliable results or conclusions; concerns about the data.

Using DM technology, this article examines the data created by platform users' actions related to rural public service and considers the future of rural public service. The following are this paper's primary innovations:

1. By using DM technology, the issues with building and running public service platforms are resolved, a personalised recommendation platform based on the platform is built, and solutions to enhance the platform's operation mechanism are offered
2. The rural public service platform based on DM provides sufficient public goods and services for the society, lays the foundation for effective social management, and maintains political stability and social development

## 2. Related Work

The public service platform involves many fields and depends on many factors, and its connotation is characterized by dynamic changes such as stages, levels, and regions. The connotation research trend of public service platform is from attaching importance to government to nongovernmental organizations, from providers to consumers, from public management to public services, and from single service to service system.

Jiang pointed out that with the emergence of the expanding government departments, the quality of public services has declined, the inefficiency of service providers, and the lack of ability to deal with the market have become increasingly prominent [10]. Zhao proposed that the government can entrust the private sector to produce and provide by means of signing contracts and granting management rights while macro-controlling public services [11]. From the perspective of consumption, Belanche analyzes two essential attributes that distinguish public goods from private goods: nonantagonistic consumption and nonexclusive consumption [12]. Perry believes that the government is a service rather than a helm. In public affairs, the needs of the people should be determined according to the will of the people. While strengthening the rights of citizens, it is emphasized that the public interest is the goal rather than a by-product. The government should provide the whole society with the public service it needs in a fair and just manner [13]. According to research by Batley et al., private competition can increase the effectiveness of public services and better safeguard customer interests [14]. Madera pointed out that privatized public service providers often ignore their social responsibilities due to the pursuit of economic interests [15]. Wu et al. proposed that government provision and private provision of services coexist, and the way of public service provision depends entirely on the quality of service that is voted by the majority [16]. Thestrup et al. also mentioned financial expenditures, paid service charges, income from drug price differences, and methods such as authorized operation, chain operation, hospital dispatch, independent operation, chain management, and group management [17, 18]. Merkel-Hess investigates the development of a rural public service platform against the backdrop of recent rural development [19].

The article "Monitoring and Path Selection of Rural Public Service Environment Based on Data Mining Technology in the New Era" was retracted in 2023. Reasons: signs of a paper mill; suspected computer-generated content; unreliable results or conclusions; concerns about the data.

Some reform recommendations are made based on the qualitative analysis of the current rural public service supply situation. They did not, however, carry out a comprehensive study of the contemporary rural public intelligence service system as a whole. Rebuilding the rural basic public service platform is more necessary given the current new situation. The basic public service platform in rural areas is explained from a theoretical standpoint in this paper. It is also examined in terms of its current issues and root causes. Based on DM technology, the paper also looks at the public service platform's user characteristics and proposes a course of action for its reconstruction. Various experiments are used to confirm the efficiency and applicability of the given strategy.

## 3. Methodology

### 3.1. Present Situation and Problems of Rural Public Services

Public services include rural public services. The government and nongovernmental public organisations and units authorised by law in the production and delivery of public goods are responsible for providing rural public service, which is a noncompetitive and nonexclusive social service [20]. Rural public service, in general, refers to the expansion of social public service into rural areas. In a limited sense, it primarily refers to the systematic and thorough management of public services offered in various fields of production and life in rural areas, based on various public services in rural areas, with rural residents and agricultural practitioners as the main service targets; At the same time, a set of all-encompassing and multilevel government public service system is established to ensure the rural economic and social development. China's rural public service system has generally made remarkable advancements throughout the years. However, the overall standard is still low, and there is a significant difference from cities. The public's social needs are diversifying as society develops, which raises expectations for both the number and quality of public services [21]. There are eight systems in the rural public service system. They are the systems for building infrastructure, extending agricultural science and technology, educating the general public, providing employment services, providing medical and health services, providing social security services, providing cultural services, and providing social management services. These eight interconnected and mutually exclusive systems make up the entire rural public service platform. In general, there are numerous causes for both the challenging transition of township government and the inadequate availability of public services in rural areas. For instance, the unjust fiscal and taxing system, the unreliable performance evaluation criteria, and so forth. The most important factor, however, is that rural public service providers are united. This is embodied in the following aspects: (1) the single supplier leads to the serious shortage of funds for public services, (2) the single supplier determines the low efficiency of the government, (3) the single supplier leads to the low quality of the staff.

The article "Monitoring and Path Selection of Rural Public Service Environment Based on Data Mining Technology in the New Era" was retracted in 2023. Reasons: signs of a paper mill; suspected computer-generated content; unreliable results or conclusions; concerns about the data.

Rural social public service availability does not currently change in response to demand. Due to the slow pace of administrative system reform and the dominance of the planning system, the provision of rural public goods is frequently influenced by higher government departments' charging and upgrading initiatives rather than local demand. The design and implementation of policies in the delivery of public services suffer from a lack of communication, and the government and farmers are unable to establish effective working relationships. In addition, due to information asymmetry, ineffective information exchange, a sluggish administrative system reform, and flawed legal system design, China's rural public services in the country's transitional period lack effective supervision. The township government has transitioned from a traditional power-based administration to a contemporary service-oriented and rule-of-law government at the same time. Higher standards for the quality of the township government workforce will undoubtedly be put forward as a result of this transition of functions. Some township government departments are accustomed to operating in accordance with the planned economic system's methods of governance, and when doing certain tasks, they frequently go above and beyond their call of duty. The majority of public servants still adhere to the regulatory government tradition instead of realising the importance of service-oriented government. Regulatory government and service-oriented government are two opposing management theories and frameworks. Most government officials do not realize these differences. The inefficiency of rural public services is mainly manifested in two aspects. First, the utilization rate of social resources is low. Second, the imbalance between supply cost and output. At the same time, rural public services have insufficient investment in education. Teachers in rural areas are very weak, and most of the education funds are raised by township governments and farmers. Compared with cities and towns, rural teachers are weak, the educational structure is single, and the educational funding gap is large. However, because of the heavy burden of education, farmers' enthusiasm for education is not high, students' enrolment rate is low, consolidation rate is low, dropout rate is high, and the number of years of education per capita is much lower than that of urban residents. In many places, nine-year compulsory education cannot be realized, and some even appear semi-illiterate. Due to the lack of state investment in rural education for a long time, coupled with the shortage of funds from the township government and farmers' income, the situation of rural education is worrying. Generally speaking, China's rural public service platform has not really been established, and there are still some problems such as insufficient supply, irrational structure, and low efficiency. At present, the singleness of the supply subject is the most fundamental reason for the difficulties in the transformation of Chinese township governments and the unsatisfactory supply of rural public services. To solve these problems, seeking multisubject supply of public services is the way out.

The article "Monitoring and Path Selection of Rural Public Service Environment Based on Data Mining Technology in the New Era" was retracted in 2023. Reasons: signs of a paper mill; suspected computer-generated content; unreliable results or conclusions; concerns about the data.

### 3.2. Construction Path of Rural Public Service Platform in the New Era

A scientific understanding of the patterns, traits, and laws governing China's economic and social growth, the scientific idea of development serves as our primary framework for completing a variety of duties at the moment. In order to give urban and rural residents, the economy, and society equal development opportunities and realise the prosperity and prosperity of the urban and rural areas, it is important to take into account the city and the countryside as a whole. Urban public facilities should be directed to cover the countryside, and modern urban civilization should spread to the rural areas. The township administration needs to modify its operations and enhance its governance structure as part of the new era's creation of rural areas. The establishment of service-oriented government objectively requires people-oriented and highlights people's people-oriented consciousness. Service-oriented government puts more emphasis on providing people with the necessary conditions or facilities on the basis of their own will. Service-oriented government not only serves some people but also provides fair, just, and satisfactory services to all people on the basis of administration according to law. At the same time, rural public service construction needs to be vigorously promoted to support the smooth development of new rural construction. Diversified public service supply is the best choice to promote the smooth realization of the two and form a benign mutual structure. In addition to the government supply system and the market supply system, bringing social organizations, especially the third sector, into the scope of system selection, and making use of the complementarity and coordination among systems to make a combination arrangement of public goods supply systems can expand the scope of system selection and search, thus making the choice of efficiency goals reliable. For the sake of morality and responsibility, the government must undertake the public service projects with pure public goods nature, which have high public welfare and lack of income, for free. The inherent attribute of public services requires the government to provide or participate in the supply of public services through fiscal expenditure, and relying on fiscal channels is an effective way to increase rural public goods. This is the main financing channel. Additionally, we can deliberately nudge social forces to deliver rural public goods via commercial channels. The development of an information publishing network should be accelerated, agricultural production should shift from one of quantity to one of quality and efficiency, and the production of agricultural products should replace the production of raw materials with the integration of production, supply, and marketing. Farmers urgently want technology for agricultural productivity, processing knowledge, and market knowledge. Creating a timely and helpful information platform and making it available to farmers for free allows them access to the network to learn about the demand and price changes of the domestic and worldwide markets for agricultural products.

The article "Monitoring and Path Selection of Rural Public Service Environment Based on Data Mining Technology in the New Era" was retracted in 2023. Reasons: signs of a paper mill; suspected computer-generated content; unreliable results or conclusions; concerns about the data.

The construction of effective supervision mechanism of rural public services is a long and complicated process. Due to the defects of current legal norms and management system, various problems are prone to occur in this project. Therefore, the government should make a good plan for the construction of rural public service supervision system from the perspective of safeguarding public interests. First, strictly control the misappropriation of public service funds. Secondly, supervision should not only be carried out within the government, but also involve the broad masses of farmers. Based on the guidance and guarantee function of policies, to improve the rural public service platform, it is necessary to take the rural economic development as the foundation, change the outdated urban-rural division policy as the starting point, strengthen the construction of relevant supporting laws and regulations, and use laws and policies to guarantee the construction of rural public service platform. Through legal means, it is necessary to formulate the law on intergovernmental relations and scientifically and rationally divide the scope of administrative and financial rights between the central government and local governments as well as between local governments. The current “top-down” decision-making system of rural public service supply is an important reason for the low efficiency of township government in providing public services. Therefore, it is necessary to change this decision-making system that determines the supply of public goods within the jurisdiction by external variables and establish a decision-making system that determines the supply of public goods within the jurisdiction. According to the nature of public goods and the characteristics of rural areas, the basic principles of promoting the construction of rural public service platform at present should be to (1) adhere to the people-oriented principle, (2) adhere to the principle of social equity, (3) adhere to the principle of classified supply, and (4) adhere to the principle of limited government. Whether the rural basic public service platform is perfect is directly related to the process of agricultural modernization, the overall development of the rural economy and the improvement of farmers' quality of life. Therefore, it is very necessary to build a perfect rural basic public service platform. This can be done from the following aspects: (1) focus on promoting the integration of urban and rural areas, (2) Increase investment in farmland water conservancy facilities, (3) continue to implement the traffic unblocked project, and (4) intensify the construction of rural electricity consumption.

### 3.3. Construction of Public Service Platform Based on DM Technology

Different definitions of DM exist. The technical definition of DM is the analysis process of employing specific technical tools to examine and process a vast amount of noisy data in order to get crucial information that humans are unaware of beforehand. DM is an interdisciplinary subject influenced by many disciplines, including database system, machine learning, statistics, visualization, and information science. From the technical point of view, it can be divided into two types: description and prediction. Among them, description refers to finding out the potential laws in data, while prediction refers to forecasting the future according to history. The main technologies commonly used in DM are artificial intelligence, database technology, and probability and mathematical statistics, especially using some mature methods and technologies in artificial intelligence. The DM process model is shown in Figure 1.

The article "Monitoring and Path Selection of Rural Public Service Environment Based on Data Mining Technology in the New Era" was retracted in 2023. Reasons: signs of a paper mill; suspected computer-generated content; unreliable results or conclusions; concerns about the data.

The iterative clustering K-Means approach is based on distance. The goal of low similarity across distinct clusters and high similarity within the same cluster can be achieved by dividing or grouping the data. From the practical point of view, DM is an iterative process. First, study the data, analyze and check the data as needed, make necessary modifications, and apply a certain method to analyze the results. Then consider these data from another angle. Then start from the beginning, use this method again or directly apply another method to get better results. Repeat for many times until the problem is solved or the desired effect appears. A very important step for DM is to recognize the purpose of DM, find out its business objects and clearly define its business problems. Although the final structure of DM cannot be predicted, the problems to be explored can be predicted. This paper mainly builds a public service platform based on DM technology.

Assuming any nonempty subset *S*⊆*L* of any frequent itemsets *L* and *L*, if:

(1) $$\begin{array}{c} \frac{\text{Support}\left(L\right)}{\text{Support}\left(S\right)}\geq \min\_\text{conf}. \end{array}$$

Then there are valid association rules:

(2) $$\begin{array}{c} R:S\Rightarrow \left(L-S\right). \end{array}$$

The confidence and support of the rule are:

(3) $$\begin{array}{c} \text{Confidence}\left(R\right)=\frac{\text{Support}\left(L\right)}{\text{Support}\left(S\right)}, \end{array}$$

(4) $$\begin{array}{c} \text{Support}\left(R\right)=\text{Support}\left(L\right). \end{array}$$

The column vector of the correlation matrix *M*_*m*×*n*_ not only represents the site structure but also reflects the common access patterns of customers; the row vector not only represents different users but also reflects the user's personalized access subgraph. Therefore, for user page clustering, the similarity of row vector and column vector can be measured separately, and the user access pattern can also be obtained by further analysis, that is, the frequent access path:

(5) $$\begin{array}{c} M_{m\times n}{\left\{\begin{array}{c} h_{11},h_{12},\cdots h_{1j},\cdots h_{1n}\\ h_{11},h_{12},\cdots h_{1j},\cdots h_{1n}\\ \cdots ,\cdots ,\cdots ,\cdots \\ h_{11},h_{12},\cdots h_{1j},\cdots h_{1n}\\ \cdots ,\cdots ,\cdots ,\cdots \\ h_{m1},h_{m2},\cdots h_{mj},\cdots h_{mn} \end{array}\right\}}_{\text{USER}}. \end{array}$$

The metric formula involved in the algorithm is as follows:

Hamming distance:

(6) $$\begin{array}{c} H_{d}\left(X,Y\right)=\overset{\left\|x\right\|}{\underset{i=1}{\sum }}\left|X_{i}-Y_{i}\right|. \end{array}$$

Among them

(7) $$\begin{array}{c} X,Y\in {\left\{0,1\right\}}^{n},n\geq 1. \end{array}$$

The threshold is

(8) $$\begin{array}{c} \Delta =2\times \overset{n}{\underset{i=1}{\sum }}\overset{n}{\underset{j=1}{\sum }}\frac{d_{ij}}{n\left(n-1\right)}. \end{array}$$

Calculate the Hamming distance between row vectors according to formula (6), and establish a distance matrix *M*_*m*×*n*_^*Hd*^ between row vectors. In a symmetric matrix *M*_*m*×*n*_^*Hd*^:

(9) $$\begin{array}{c} d_{ij}\in M_{m\times n}^{Hd}\left(1\leq i\leq m,i<j\leq n\right). \end{array}$$

Among them, *d*_*ij*_ represents the Hamming distance between the *i* and *j* row vectors. Standardize the data in the decision matrix, and the calculation formula of the standardized attribute value *r*_*ij*_ is:

(10) $$\begin{array}{c} r_{ij}=f_{ij}/\sqrt{\overset{m}{\underset{i=1}{\sum }}{f_{ij}}^{2}},i=1,2,3,\cdots ,m;j=1,2,3,\cdots ,n. \end{array}$$

Compute the weighted normalized decision attribute value *v*_*ij*_:

(11) $$\begin{array}{c} v_{ij}=w_{j}r_{ij},i=1,2,3,\cdots ,m;j=1,2,3,\cdots ,n. \end{array}$$

Here *w*_*j*_ is the relative weight of the *j* attribute or indicator, and ∑_*j*=1_^*n*^*w*_*j*_ = 1. The limited public service resources with a total amount of *R* are allocated through the *n*line, and the consumer will choose a certain channel to receive the service according to their own situation. According to the evaluation and behavior selection results of the consumer subjects, the large-scale consumer subjects are divided into *n* relatively small groups to gather:

(12) $$\begin{array}{c} g_{j},j\in \left(1,\cdots ,n\right). \end{array}$$

The corresponding group size is *c*_*j*_. There are *m* allocation schemes:

(13) $$\begin{array}{c} a_{i},i\in \left(1,\cdots ,m\right). \end{array}$$

The resource allocation matrix is:

(14) $$\begin{array}{c} A={\left\lfloor a_{ij}\right\rfloor }_{m\times n}. \end{array}$$

Among them, ∑_*j*=1_^*n*^*a*_*ij*_ = *R*, the resource allocated to group *g*_*j*_ by scheme *a*_*i*_ is *a*_*ij*_.

The article "Monitoring and Path Selection of Rural Public Service Environment Based on Data Mining Technology in the New Era" was retracted in 2023. Reasons: signs of a paper mill; suspected computer-generated content; unreliable results or conclusions; concerns about the data.

The public service platform is B/S database application system software. This paper designs and implements a DM system integrated under this platform, so the platform is designed based on B/S framework. Part of the mining data storage is different from the original way. The “platform” retrieval uses the search of index layer to generate results, while both the mining object data and the result data are stored in the database.  Figure 2 shows the acquisition and transmission function module.

Before the system scans, the database must be sorted out and unnecessary transactions deleted so as to reduce the scanning workload and improve the work efficiency. At the same time, when selecting candidate sets, select candidate sets with fewer elements as much as possible, that is to say, delete some attributes before selecting, so as to reduce the system overhead. The public service platform supports users to upload data files and select the data attribute fields in the data files as data analysis objects. By reading all attribute fields in the data set, users can analyze the data set between any attributes. In the process of platform operation, DM technology is adopted to provide and demand the nature and service of CAD/CAE resources for users, the CAD/CAE service between users and service organizations, and the interactive service chain between users and platform subsystems. Through data collection, data processing, data storage, and pattern discovery, useful patterns are found and various mechanisms of the platform are adjusted.

## 4. Result Analysis and Discussion

Areas A and B, two exemplary cities, are chosen as the experimental objects in this paper. In the experiment, 254,637 pieces of data were mined in area A while 305,487 pieces were mined in area B. The data analysis algorithm, which is directly related to the analysis tasks supplied by users, the parameters of the algorithm, the preprocessing of the data, and other entities, forms the basis for the design and implementation of the platform. Data conversion: convert the experimental data from csv file format to arff file format. In addition, association rules can only deal with the situation that all attributes are classified. At this time, the numerical attribute is discretized. The data cleaning stage mainly completes the data row dimension reduction and column dimension reduction. Dimension reduction is mainly to delete rows according to the conditions of cleaning rule base. Dimension reduction refers to keeping the required attribute columns according to the mining task. The data selected in the experiment have the same identity repeated at different times, and the number of such repeated occurrences can be understood as someone's support in the data set. The hardware requirements of this system are general, only a few dual-core machines are needed. Choose the computer with better performance as the DM server for analyzing the characteristics of users, and other computers are used by users. Users can access the web pages in the network to generate access data for testing and store them in the system. The specific development environment is shown in Table 1.

The article "Monitoring and Path Selection of Rural Public Service Environment Based on Data Mining Technology in the New Era" was retracted in 2023. Reasons: signs of a paper mill; suspected computer-generated content; unreliable results or conclusions; concerns about the data.

During the mining process, the platform needs to frequently compare the exchange identification, and there are many digits of ID number and passport number. Therefore, in order to simplify the calculation in the mining process, the platform replaces the unique identification of personnel with a short combination of letters and numbers. In this paper, by setting the extended attribute of IIS log and using Cookie technology, adding the reading and writing operation of user's Cookie in IIS, the user's Cookie log can be written into the extended attribute of Web log of the server. When users visit IIS, a public service platform, there will be Cookie attributes that record users. If the Cookie is deleted or invalid, it means that a new user is accessing it. The training curve of the algorithm is shown in Figure 3.

In this study, the user interface reads the data file's selected data attribute column information to allow users to choose attribute fields. Then, with the help of the public service platform's database table, the variables and parameters of the chosen analysis algorithm are provided, and the parameter variable values are saved in the database table through the user interface settings and sent to the corresponding data analysis algorithm. The experimental outcomes demonstrate that the algorithm's mistake is depicted in Figure 4.

There are many factors that can affect the mining results in the whole implementation process of the mining platform, including the data itself, the granularity and span definition of transaction database and the selection of mining parameters. Different settings of parameter values in the algorithm and different data processing situations may cause a big deviation in the results. The following is the analysis of mining parameters. Set |*R*| as the number of all frequent sets, and |*R*′| as the number of frequent sets with abnormal looseness.  Figure 5 shows the variation of |*R*′|/|*R*| with the minimum support parameter.

Mining those association rules with support between 10% and 100%, lift value over 1.5, and lift value in the top 100. First, the user inputs the minimum support and confidence, and the platform implements mining. The minimum support of the experiment is 2, and the minimum confidence is 35%. If the users who exceed the minimum support count have visited all the pages in a certain group of pages in one visit transaction, this group of pages is called a group of pages. These web page groups reflect the relevance of different pages being visited by a certain number of users. After the experiment, this paper obtains the statistics as shown in Table 2.  Table 3 is the comparison table of frequent sets of abnormal looseness.

The article "Monitoring and Path Selection of Rural Public Service Environment Based on Data Mining Technology in the New Era" was retracted in 2023. Reasons: signs of a paper mill; suspected computer-generated content; unreliable results or conclusions; concerns about the data.

The establishment of a good transaction database can not only improve the execution time of subsequent Web log mining algorithms but also improve the response speed of the platform. In this paper, the response speed of different algorithms is tested, and the results are shown in Figure 6.

Data analysis is a purposeful and organized process of collecting data, analyzing it, and converting it into information. This paper obtains the user characteristics through data analysis. By using the function of personnel relationship analysis of the platform, the platform can obtain the background relationship weights of the specified data sets in the whole database. The size of the data sets is limited to a certain extent, generally no more than 10 items. The platform has the function of personnel relationship analysis and provides data interface to external programs. The interface contains several parameters as follows: personnel number, personnel ID queue, data source and retrieval level.  Figure 7 shows the accuracy of the user characteristics obtained by algorithm analysis.

This part chooses data from two locations for mining experiments, examines the results of the experiments in light of the actual company operations, and examines the variables that may influence the mining outcomes. According to experimental findings, this method is 94.38% accurate. This technique can efficiently mine user characteristics and offer technical assistance for modern rural public services.

## 5. Conclusion

Enhancing the development of rural public service platforms is a fundamental prerequisite for creating an overall prosperous and peaceful society. The goal of this article is to explain how to create a platform for rural public service in the new era and present the route that rural public service should take. Based on this, this article creates and implements a public service platform based on DM technology, fuses the actual job requirements with DM technology, and analyzes vast amounts of basic data in an effective attempt to use mining to resolve real-world business issues. In order to offer some support in the decision for the choice of path for rural public service in the new era, this article simultaneously examines the realistic predicament of rural public service and, based on DM technology, digs the user characteristics of public service platform. This study then chooses data from two locations for mining experiments, analyzes the experimental findings in light of real-world company operations, and examines the variables that may influence the mining outcomes. According to experimental findings, this method is 94.38% accurate. This technique can efficiently mine user characteristics and offer technical assistance for modern rural public services. However, the public service platform does not perform additional support or conditional judgement for the initial data set uploaded by users, necessitating more development in subsequent work when the public service platform interfaces with the analysis algorithm.

The article "Monitoring and Path Selection of Rural Public Service Environment Based on Data Mining Technology in the New Era" was retracted in 2023. Reasons: signs of a paper mill; suspected computer-generated content; unreliable results or conclusions; concerns about the data.

## Figures and Tables

**Figure 1:** DM process model.

**Figure 2:** Acquisition and transmission function module.

**Figure 3:** Training curve of algorithm.

**Figure 4:** Error curve of algorithm.

**Figure 5:** |*R*′|/|*R*| changes with the minimum support parameter.

**Figure 6:** Response speed curves of different algorithms.

**Figure 7:** Accuracy of user characteristics obtained by algorithm analysis.

**Table 1:** Platform development environment.

Operating system	Linux
Database	MySQL
Development tools	Eclipse
Development language	Java
System software	jdk1.6, MySQL, eclipse

**Table 2:** Comparison table of frequent sets with confidence greater than 35%.

	Support degree	Frequent set	Quantity
H	2	C2	17214
		C3	3657
		C4	601
		C5	36
	3	C2	3208
		C3	218
		C4	15
	4	C2	168
		C3	25
	5	C2	128

X	2	C2	19654
		C3	3021
		C4	1637
		C5	101
	3	C2	3411
		C3	435
		C4	28
	4	C2	78
		C3	16
	5	C2	241

**Table 3:** Comparison table of abnormal looseness frequent set.

	Support degree	Frequent set	Quantity
H	2	C2	142
		C3	38
		C4	6
		C2	38
		C3	15
		C4	5
		C2	11
		C3	4
		C2	4

X	2	C2	121
		C3	27
		C4	9
	3	C2	18
		C3	12
		C4	11
	4	C2	16
	5	C2	2

## Data Availability

The data used to support the findings of this study are available from the corresponding author upon request.
